The article "The Efficacy of Rehabilitation Nursing Interventions on Patients with Open Lower Limb Fractures" was published in 2022. Journal: J Healthc Eng.

# The Efficacy of Rehabilitation Nursing Interventions on Patients with Open Lower Limb Fractures

**DOI:** 10.1155/2022/1859747

**Published:** 2022-04-16

**Authors:** Zengfen Pang, Meimei Shan, Yuanyuan Li, Huan Zhang, Amei Huang, Yuping Liu, Xianghong Li

**Affiliations:** ^1^The Affiliated Cancer Hospital of Shandong First Medical University, Jinan, Shandong, China; ^2^Chinese Nursing Society, Beijing, China

## Abstract

**Objective:**

The study aims to analyze the efficacy of rehabilitation nursing interventions on patients with open lower limb fractures.

**Methods:**

From June 2020, patients who received RNI (observation group) were included and compared with patients who received routine nursing interventions (control group). The efficacy of different nursing modes was compared with several indicators.

**Results:**

One hundred patients were included in this study, 50 in each group. The baseline characteristics were not significantly different between the groups. Regarding the emotional scores, the Self-Rating Anxiety Scale (SAS) score (26.98 vs 43.47), and Distress Management Screening Measure (DMSM) score (8.01 vs 12.85) in the observation group were significantly lower than those in the control group, both *P* < 0.05. Regarding the postoperative related indexes, the postoperative pain score (10.13 vs 15.53), fracture healing time (6.32 vs 10.86 weeks), and postoperative complications rate (0 vs 12%) in the observation group were all significantly lower than those in the control group, all *P* < 0.05. Regarding the quality of life scores, the WHOQOL-100 score (94.12 vs 83.13) and PSQI score (6.43 vs 10.36) were both significantly better in the observation group, with both *P* < 0.05.

**Conclusion:**

Patients with open lower limbs who received RNI can help patients reduce postoperative anxiety and stress, promote postoperative rehabilitation and improve their quality of life.

## 1. Introduction

With the rapid development of China's construction industry and transportation industry, the incidence of open fractures of the lower limbs is also increasing year by year. The trauma caused by the fracture is large. Serious conditions such as tissue defects, bone fracture exposure, and wound infection may occur in these kinds of fractures, resulting in aggravating the pain of patients and delaying their postoperative recovery [1]. Even physical and psychological stress responses will occur in these patients [2].

In order to further reduce the complications and promote the recovery of lower limb function, it is necessary to find scientific measures for patients with open lower limb fractures. Researchers have identified the positive clinical value of rehabilitation nursing interventions (RNI) in patients who underwent general surgeries and orthopedic surgeries [3, 4]. The postoperative RNI may play an important role to ensure the quality of rehabilitation. However, studies about the efficacy of RNI on patients with open lower limb fractures are still rare. Therefore, we conducted a retrospective case-control study to explore the efficacy of RNI compared with routine nursing interventions, and the content is further discussed in this study.

## 2. Methods

The RNI was adopted in our department since 2020 June. The patients who received RNI after 2020 June were included in our study.

### 2.1. Case Selection Criteria

#### 2.1.1. Inclusion Criteria

The inclusion criteria were as follows: (1) detailed imaging data can be obtained; (2) age ≥18 years old; (3) meet the standards of surgical operation and anesthesia; (4) has no treatment contraindications and midway withdrawal; (5) normal coagulation function, cardiopulmonary, liver, and kidney functions; and (6) patients or family members were aware of the study and signed the consent [5].

#### 2.1.2. Exclusion Criteria

The exclusion criteria were as follows: (1) minors; (2) women in pregnancy and lactation; (3) with emotional and mental disorders; (4) with other fractures; (5) with blood disease; and (6) patients with malignant tumors [6].

### 2.2. Nursing Methods

Patients in the control group were given routine nursing and the corresponding nursing and guidance according to the patient's situation. Patients in the observation group provided RNI, the details are further discussed in this study [7].

#### 2.2.1. Evaluation

The postoperative rehabilitation plan was conducted based on the data after a comprehensive examination of the patient's postoperative situation. Communication was strengthened to help patients improve their negative postoperative emotions. Nurses gave targeted nursing interventions for common postoperative complications. The patient's body position was adjusted in time. It is recommended to rest in a rigid bed within 3 weeks after surgery and turn over once every 2 hours. Family members were taught to massage their limbs to effectively prevent pressure sores. Good pain management was carried out for patients to relieve postoperative pain. If the patient took a flat rest, the elbow was extended with a back flexion of 30–40°. When taking the side position, the lower limb's joints were slightly flexed to avoid compression of the upper limbs. Some patients had obvious pain due to their own tolerance, and painkillers were taken under the guidance of the attending doctor to relieve the pain when necessary. When the patient was in pain, the pain pump was used to maximize the pain caregivers' acceptance of the patient. The patient was informed of the attention of the matters in the recovery process. The pain management methods and rehabilitation knowledge were explained, rehabilitation guidance and training were appropriately strengthened, and the patient's immunity was improved [8].

#### 2.2.2. Psychological Nursing Care

Patients with an open fracture of the lower limbs often have severe pain after surgery, leading to a serious bad mood. This kind of bad mood is different from the concerns about surgery preoperatively. Therefore, the psychological counseling strategy adopted by nurses postoperatively is different from that of preoperatively. The proper pain relief guidance and detailed health education were based on timely counseling on patients' physical discomfort and pain condition. Nursing staff should communicate with patients actively to tell them the importance of postoperative medical and nursing cooperation. As a result, the patients' own medical compliance behavior was strengthened [9].

#### 2.2.3. Pain Care

Nursing staff should determine the degree of postoperative pain and analyze the impact of pain symptoms on the quality of sleep.

In order to avoid the use of analgesics, nursing staff should explain how to divert pain attention to patients when the pain can be tolerated. The nursing staff were required to strengthen ward inspection [10] to inquire about the pain degree every day. If the VAS score exceeds 4 points, then report the pain to the doctor in time. After the feedback from the doctors, nursing staff should follow the doctor's advice to provide pain treatment if necessary.

#### 2.2.4. Health Education

Nursing staff should explain the necessity of postoperative rehabilitation care, the high-risk factors that affect postoperative recovery, and the ways of postoperative rehabilitation care. Online consultation was also available for patients to clear up their doubts about the diseases and surgical treatment.

Nursing staff should guide the daily lives of patients to balance bed and activity. Exercise is necessary as soon as possible after the operation to promote blood circulation in the lower limbs. The amount of activity can be gradually increased according to the needs of rehabilitation and the condition of pain. Patients were advised to eat foods with high energy to promote the recovery of wounds. Smoking and drinking were forbidden during the rehabilitation period, and drinking more water was encouraged [11].

#### 2.2.5. Prevention of Postoperative Complications

During the period of an indwelling catheter, nurses should carry out bladder training for the patient to prevent bladder muscle atrophy. After the patient's postoperative condition went well, intermittent catheterization was used to continuously strengthen its own urination function.

Nurses were required to advise patients and their family members of the guidance to avoid wound infection. The prevention methods include disinfecting and cleaning the pressed skin, informing patients not to scratch the wound with their hands, treating timely when the wound was contaminated by blood, and maintaining the skin dry.

There are four aspects to do a good job in the prevention of deep vein thrombosis (DVT). First of all, intravenous care. In order to prevent DVT, lower extremity puncture and infusion are avoided, especially repeated operations at the same location. When infusing drugs, the doctor's advice is followed to choose less irritating drugs for the patient to prevent the liquid from leaking out of the blood vessels. When using a touquet, it is necessary to reduce the binding time to avoid unnecessary damage to the distal and local blood vessels. The puncture site is closely observed, the inflammatory reaction is found and dealt with in time, and the venous channel is reselected. Secondly, lower extremity care. In order to effectively prevent deep venous thrombosis of the lower extremities, nurses instructed patients to raise the affected limb after surgery to facilitate the venous return of the lower extremities and prevent swelling. It should be careful not to compress the deep veins of the patient's legs. The color and temperature of the affected limb were observed, and the pulse of the dorsal foot artery was accurately recorded. On this basis, the cause of the abnormality in time was found and dealt with accordingly. When necessary, an intermittent inflation and compression device were used to perform periodic compression to improve the venous blood flow of the lower extremities and prevent deep vein thrombosis in the lower extremities. At the same time, medication guidance for patients with severe renal insufficiency or patients with thrombosis, unfractionated heparin can be used. The specific dosage depends on individual differences. The patient needs to be continuously monitored for coagulation indicators during the medication process to avoid medication risks. Low-dose heparin has a good effect of preventing thrombosis. It is recommended to use 5000 U subcutaneous injection 2 h before the operation and to monitor the patient's platelet function after the operation to avoid thrombocytopenia. Finally, mechanical prevention. Medical elastic stockings are used to apply external force to restrict venous pressure, promote venous return, and ensure the normal blood circulation function of the veins of the lower extremities, thereby exerting a preventive effect. At the same time, the use of intermittent inflation and compression devices to periodically pressurize patients can also improve the venous blood flow of the patients' lower limbs, increase blood flow, and prevent DVT [12].

#### 2.2.6. Rehabilitation Guidance

1. Passive training program. After the operation, a rehabilitation training program was developed for the patient based on the preoperative examination results and the postoperative condition. On the first postoperative day, the patient's affected limb was properly raised and kept in a straightened state to avoid external rotation, and the patient's pain symptoms were evaluated. Patients were encouraged to take the initiative in bed activities. When the patient's pain is mild, their knee joints were passively moved, and ankle back extension exercises and quadriceps isometric exercise training were performed. Patients were instructed to perform ankle pump exercises and quadriceps contraction training to enable patients to master the essentials of movement to accelerate venous return. The patient was instructed to train for muscle tension and contraction. The affected limb was raised by 20∼30°. Passive activities should be based on the comfort of the patient. Pillows were not put under the knees, letting the patients raise their entire lower limbs, and placing hard objects under the knees was avoided to avoid hitting the popliteal veins. Oppression was produced. Patients were instructed to press and rub the muscles of the lower limbs at the base of their palms to speed up blood flow, promote venous return, and prevent thrombosis. Patients were instructed to raise their straight legs, exercise their muscles, and prepare themselves for getting out of bed later. The condition of the dorsal artery of the device was closely observed to determine the degree of swelling of the limbs. If there was any abnormality, it was immediately notified to the doctor. On the 3rd day after the operation, the patient's knee joint passive training was carried out with the aid of the joint continuous passive activator. On the 4th to 7th day after the operation, the patient was given quadriceps isometric contraction exercise training, straight leg raising exercise training, and active knee flexion exercise training [13].
2. Active training program: elastic bandages should be used when the patient goes down to the ground to reduce edema of the lower extremities, speed up the return of venous blood, and avoid thrombosis. According to the patient's postoperative recovery, the patient is guided to restore and contract the quadriceps, ankle joint, and gluteal muscles to avoid complications such as osteoporosis, venous thrombosis, and muscle atrophy. The changes in the recovery of the disease are observed, the patient's hip and knee joint flexion and extension strengths are trained in a timely manner, and the activities of the upper and lower joints of the fracture are carried out. According to the patient's recovery degree, the activity intensity can be appropriately increased to improve joint stiffness. Nursing staff should regularly perform related passive activities for the patient, and then gradually change to active activities, allowing the patient to lie on the bed to perform active leg elevation exercises, and assist them to restore their sitting ability until they can walk slowly and stand up. When the patient can stand autonomously and the affected leg can move forward, walking training is started. Limbs, standing, striding, and other exercises are guided, the patient's gait is observed, a walker is used to assist walking training at an appropriate time, or a small amount of support from family members is provided. Early walking training needs to pay attention to that the amount of activity should be moderate to avoid foot varus, and the patient is required to use the affected side of the lower limb to shift the center of gravity, and the healthy side of the lower limb cannot be used to help walk, to avoid gait instability, and to prevent the occurrence of spasm of the affected side of the lower limb. The range of movement of the uninvolved limb of the patient is controlled, requiring the patient not to move the uninhibited limb at will during training but to use the affected limb subconsciously [14].

### 2.3. Observation Indicators

The anxiety scores before and after nursing were compared using the Self-Rating Anxiety Scale (SAS). The critical value is 50 points: (1) mild anxiety: 50–59 points; (2) moderate anxiety: 60–69 points; and (3) severe anxiety: >69 score [8]. The psychological pain scores before and after the intervention were compared using the distress management screening measure (DMSM) scale; 0–10 points, 0 points for no psychological pain, and 10 points for extreme psychological pain [9]. The postoperative pain scores, fracture healing times, and times of the two groups of patients postoperative complications were compared. The quality of life scores of the two groups of patients before and after intervention were compared using the World Health Organization Quality of Life Scale (WHOQOL-100 scale). There are a total of 25 subitems. Each subitem is evaluated according to the 0–4 point method. The total score is 100 points. The higher the score, the higher the quality of life. The comparison of the sleep quality scores of the two groups of patients before and after intervention, using the Pittsburgh Sleep Quality Index (PSQI) scale, 7 evaluation items, 0–3 points scoring method, a total score of 21 points; the lower the score, the better the sleep quality [15].

### 2.4. Statistics

In this study, SPPS20.0 was used for statistical analysis. The measurement data were described by the mean ± standard deviation ($\bar{x}\pm s$), and student's *t* test was used; the count data were described by example (%), and the *χ*^2^ test was used. *P* < 0.05 means that the difference is statistically significant.

## 3. Results

### 3.1. Baseline Characteristics

In this study, 100 patients were included in this study. In the observation group, 50 patients with open lower limb fractures were included with men: women as 29 : 21. The mean age was 41.89 ± 1.38 years (a range of 25–70 years). The causes of fracture were as follows: 37 traffic accidents, 10 high falls, and 3 other causes. The fracture areas were as follows: 28 femur and 22 tibia. Fracture Gustilo–Anderson classification: 44 A and 6 B. In the control group, there were 32 men and 12 women aged 23–70 years on average (42.71 ± 1.29). Fracture causes were as follows: 34 traffic accidents, 12 falling injuries, and 4 other cases. The fracture areas were as follows: 30 femur and 20 tibia. Fracture Gustilo–Anderson classification: 42 A and 8 B. The two general data comparison results were *P* > 0.05, comparable.

### 3.2. Effects of RNI on Postoperative Emotional Scores

The comparison of SAS score (64.12 vs 64.30) and DMSM score (17.32 vs 17.46) had no significant difference between the two groups before nursing, with both *P* > 0.05. After the nursing intervention, the scores significantly improved compared with the same group before nursing, *P* < 0.05. Moreover, after the intervention, the abovementioned scores in the observation group decreased significantly more than in the control group (26.98 vs 43.47 and 8.01 vs 12.85), both *P* < 0.05 (Table 1).

### 3.3. Effects of RNI on Postoperative Related Indexes

The postoperative pain score (10.13 vs 15.53) and fracture healing time (6.32 vs 10.86 weeks) of the observation group were lower than those of the control group, *P* < 0.05; postoperative complications (0) in the observation group were lower than those of the control group (12.0%), *P* < 0.05 (Table 2).

### 3.4. Effects of RNI on Postoperative Life Quality Scores

The comparison of WHOQOL-100 scores and PSQI scores between the two groups before nursing had no significant difference with *P* > 0.05. After the nursing intervention, the PSQI score of the observation group was lower than that of the control group (94.12 vs 83.13), and the WHOQOL-100 score (6.43 vs 10.36) was higher than that of the control group with both *P* < 0.05 (Table 3) [13].

## 4. Discussion

Open fracture of the lower limbs is a common type of fracture in clinic practice, which can seriously damage the walking function and affect the daily life of patients. Although aggressive surgical strategies will be adopted, limb dysfunction will still occur in some patients. Moreover, the high risk of infection and strong traumatic stress response of patients was also associated with this kind of fracture [16]. Therefore, it is the common pursuit of orthopedic researchers to take effective measures to promote the prognosis of patients with lower limb fractures.

The concept of rehabilitation nursing focuses on applying multidisciplinary theories to formulate targeted treatment measures to reduce the psychological and physical stress and trauma caused by surgical operations on patients and to promote rehabilitation. [15] The efficacy of RNI has been identified in many fields. However, there is no systematic and authoritative research data about the efficacy of RNI in patients with open low limb fractures. Therefore, we conducted this study because we hypothesized that RNI may be helpful in improving the prognosis of patients with open low limb fractures. Finally, we identified that RNI can help patients reduce postoperative anxiety and stress, promote postoperative rehabilitation, and improve quality of life.

The psychological impact of open fracture surgery on patients is relatively large. Unhealthy emotions such as worry, anxiety, and depression may come from the burden of disease and economic conditions. The unhealthy emotions may decrease compliance and finally worsen the prognosis. Integrating postoperative psychological care into RNI is a supplementary nursing model for humanized nursing intervention. The model aims to help patients overcome their inner conflicts through communication and opinion exchanges. In previous studies, psychological nursing has been identified as playing an important role in the recovery of patients after surgery and in some chronic diseases. [17, 18] In our study, we also found emotional scores significantly improved after psychological nursing intervention in patients with open lower limb fractures.

Postoperative pain is a common phenomenon that often occurs within 3 days after an operation, and the incidence rate is as high as 95%. It is the result of the combined effects of fracture pain, surgical pain, postoperative swelling, and compartment syndrome. Severe pain after fracture is a malignant stimulus, which can cause severe pain stress damage and traumatic pathological changes, such as increased systemic oxygen consumption, decreased body immunity, metabolic disorders, rapid loss of nutrients, high blood pressure, and shock response. It will damage the functions of various systems of the human body and affect the postoperative rehabilitation effects [19, 20]. Therefore, improving postoperative pain in patients with open lower limb fractures is of great significance for promoting postoperative recovery. The results of this study showed that RNI can significantly reduce the degree of postoperative pain in patients with open lower limb fractures.

Postoperative DVT is a common complication after surgery for open fractures of the lower limbs. It is generally recognized that early functional exercises and activities can reduce the incidence of postoperative complications [21]. Moreover, DVT can be prevented by many nursing interventions. In the conventional nursing mode, activities are restricted in the early stages after the operation. After the pain is relieved, the patient is encouraged to exercise moderately, but no specific requirements are made to avoid unnecessary trauma, which increases the risk of complications. RNI advocates early activities to avoid DVT caused by blood circulation disorders in the lower limbs. Therefore, DVT can be prevented by RNI [22]. The effects of RNI were identified in our study.

The quality of life and quality of sleep are very important evaluation indicators. Due to the reduced postoperative pain and complications, the WHOQOL-100 score and PSQI score improved significantly. The use of RNI is beneficial to the improvement of the quality of life and quality of sleep of patients with open lower limb fractures.

Our study had several limitations worth discussing. First, its retrospective nature prevented us from making stronger conclusions. The second limitation was the small sample size. Due to RNI being adopted in our hospital less than 2 years, the accumulated cases were not common in our center. Third, a lack of objective indicators may cause bias. More multicenter prospective studies with a large sample size are necessary to better understand the true value of RNI.

## 5. Conclusion

Based on a retrospective case-control study, we identified that patients with open lower limbs who received RNI can help reduce postoperative anxiety and stress, promote postoperative rehabilitation, and improve quality of life. More multicenter prospective studies with a large sample size are necessary to better understand RNI. More multicenter prospective studies with a large sample size are necessary to better understand the true value of RNI.

## Figures and Tables

**Table 1:** Comparison of emotional scores between the two groups before and after nursing intervention $\left(\bar{x}\pm s\right)$.

Group	SAS score (points)		DMSM score (points)	
	Before intervention	After the intervention	Before intervention	After the intervention
Observation group (*n* = 50)	64.12 ± 5.63	26.98 ± 2.12^*∗*^	17.32 ± 1.25	8.01 ± 0.31^*∗*^
Control group (*n* = 50)	64.30 ± 5.71	43.47 ± 3.41^*∗*^	17.46 ± 1.33	12.85 ± 1.68^*∗*^
*t* value	0.569	12.489	0.651	11.824
*P* value	0.239	0.000	0.304	0.000

Note: comparison results of before and after interventions within the group, ^*∗*^*P* < 0.05; SAS = Self-rating Anxiety Scale; DMSM = distress management screening measure.

**Table 2:** Comparison of related indicators between the two groups before and after nursing intervention $\left(\bar{x}\pm s\right)$.

Group	Pain score (points)	Fracture healing time (weeks)	Postoperative complications, *n* (%)
Observation group (*n* = 50)	10.13 ± 0.46	6.32 ± 0.33	0 (0)
Control group (*n* = 50)	15.53 ± 1.13	10.86 ± 0.78	6 (12.0)
*t* value	9.637	8.561	8.356
*P* value	0.000	0.000	0.008

**Table 3:** Comparison of sleep and quality of life scores between the two groups $\left(\bar{x}\pm s\right)$.

Group	WHOQOL-100 score (points)		PSQI score (points)	
	Before intervention	After the intervention	Before intervention	After the intervention
Observation group (*n* = 50)	78.24 ± 3.63	94.12 ± 2.69^*∗*^	14.32 ± 1.25	6.43 ± 0.12^*∗*^
Control group (*n* = 50)	77.92 ± 3.77	83.13 ± 3.24^*∗*^	14.46 ± 1.33	10.36 ± 0.68^*∗*^
*t* value	0.639	13.826	0.639	15.278
*P* value	0.207	0.000	0.591	0.000

Note: comparison results of before and after interventions within the group, ^*∗*^*P* < 0.05; WHOQOL-100 = World Health Organization Quality of Life Scale; PSQI = Pittsburgh Sleep Quality Index.

## Data Availability

All the data generated or analysed during this study are included in this article.
